# A New Implementation of Genome Rearrangement Problem

**DOI:** 10.1155/2021/6692775

**Published:** 2021-01-23

**Authors:** Xiaoqian Jing, Haihe Shi

**Affiliations:** School of Computer and Information Engineering, Jiangxi Normal University, Nanchang 330000, China

## Abstract

Unsigned reverse genome rearrangement is an important part of bioinformatics research, which is widely used in biological similarity and homology analysis, revealing biological inheritance, variation, and evolution. Branch and bound, simulated annealing, and other algorithms in unsigned reverse genome rearrangement algorithm are rare in practical application because of their huge time and space consumption, and greedy algorithms are mostly used at present. By deeply analyzing the domain of unsigned reverse genome rearrangement algorithm based on greedy strategy (unsigned reverse genome rearrangement algorithm (URGRA) based on greedy strategy), the domain features are modeled, and the URGRA algorithm components are interactively designed according to the production programming method. With the support of the PAR platform, the algorithm component library of the URGRA is formally realized, and the concrete algorithm is generated by assembly, which improves the reliability of the assembly algorithm.

## 1. Introduction

With the development of biotechnology, biological information data is growing explosively. At the same time, the improvement of computer computing ability and the development of Internet make it possible to store and process large-scale data. How to use computer technology to extract useful information from these data is imminent. Therefore, bioinformatics emerges as the times require. Bioinformatics covers the comprehensive application of biology, computer science, and mathematics. Through the collection, processing, storage, dissemination, analysis, and interpretation of biological information, the biological significance of a large amount of data is clarified and understood.

In organisms, a chromosome is composed of a gene sequence, and the genome is a collection of chromosomes [1]. In order to determine the similarity or homology between the two organisms and reveal the problems of biological heredity, variation, and evolution, we often arrange and compare the two DNA sequences of two organisms according to certain rules. Then, through a series of basic operations such as character editing (insert, delete, and replace), one sequence is transformed into another. The minimum number of editing operations required to complete this conversion is the edit distance of two sequences. At the level of a single gene, genetic sequences evolve by editing these characters, so edit distance is a useful measure of evolutionary distance. However, at the chromosomal level, genetic sequences are mainly evolved by global genome rearrangements. There are five basic rearrangements, namely, translocation, transposition, duplication, deletion, and reversal. Translocation refers to the partial exchange of two nonhomologous chromosomes in a genome. Translocation refers to the exchange of two contiguous gene subsequences in a chromosome. Replication refers to the replication of a continuous gene subsequence on a chromosome. Deletion refers to the deletion of a continuous gene on a chromosome, and inversion refers to the sequence reversal of a continuous gene on a chromosome. Inversion is the most common of these five forms, especially in organisms with only one chromosome. For example, the only difference between the gene sequences of the two most famous bacteria, *Escherichia coli* and *Salmonella typhimurium*, is the inversion of a subsequence of the chromosome sequence [2]. In the fruit fly, genus *Drosophila*, inversion can reflect the differences between species and within species more frequently than translocation or other processes [3]. In these examples, the importance of inversion shows that the research on the algorithm of genome rearrangement only by inversion (we call it reverse genome rearrangement) is a valuable step to study the evolutionary distance at the chromosome level.

In this paper, we design an abstract generic algorithm component library of unsigned reverse genome rearrangement algorithm (URGRA) based on greedy strategy, which improves the reliability and reusability of algorithms in this field. The second section introduces the genome rearrangement problem and related research and briefly describes the domain modeling technology and formal methods. The third section analyzes the domain of reverse genome rearrangement algorithm domain, establishes the domain feature model of URGRA, identifies the common features and variable features, establishes the relationship between features, and designs algorithm components and component interaction model. In Section 4, we show the process of developing a reverse sorting algorithm based on the First Descending Strip Reversal (FDSR) based on the component library and give the experimental results of the algorithm. Finally, we summarize and prospect the full text.

## 2. Materials and Methods

### 2.1. Reverse Genome Rearrangement Problem

Given two chromosomes, they are represented by *τ* and *σ*, respectively, *τ*=*τ*_1_, *τ*_2_, *τ*_3_,…, *τ*_*n*_, *σ*=*σ*_1_, *σ*_2_, *σ*_3_,…, *σ*_*n*_, where *σ*_i_ and *τ*_i_ represent a gene on the chromosome, and let *ρ* *=* [i, j] (1 ≤ *i* ≤ *j* ≤ *n*) denote the inversion interval acting on the chromosome. *σ·ρ* denotes that the subsequence [*σ*_*i*_, *σ*_*i*+1_,…, *σ*_*j*−1_, *σ*_*j*_] in *σ* is transformed into [*σ*_*j*_, *σ*_*j*−1_,…, *σ*_*i*+1_, *σ*_*i*_].

What we want to seek is the minimum value of inversion operation; that is, to find a series of inversion interval *ρ*_1_, *ρ*_2_, *ρ*_3_,…, *ρ*_r_ makes *σ·ρ*_1_*·ρ*_2_*·ρ*_3_…*ρ*_r_ = *τ* and *r* is the smallest. We call *r* the reverse distance or inversion distance of *σ* and *τ* and record it as *d*_(*σ,π*)_ (although it cannot guarantee that the inversion process represents an actual evolutionary sequence, it can give us a lower bound of the number of rearrangements that have occurred and indicate the similarity between two species. Therefore, scientists are interested in the minimum number of reversals [4]).

For the convenience of research, we use the natural number to represent each gene from the mathematical point of view; that is, given a sequence *τ*=(*τ*_1_, *τ*_2_, *τ*_3_,…, *τ*_*n*_), the number *Z* is used to represent *τ*_z_ (*z* = 1, 2, 3,…, *n*). By multiplying *τ*^*−1*^ at both ends of *σ·ρ*_*1*_*·ρ*_*2*_*·ρ*_3_…*ρ*_r_ = *τ*, we can get the expression *τ*^*−1*^*·σ·ρ*_1_*·ρ*_2_*·ρ*_3_…*ρ*_r_ = *l*, *l* is expressed as the identity arrangement (i.e., the sequential arrangement of natural numbers 1, 2, 3, ..., *n*), and *τ*^*−1*^ is the inverse of permutation *τ* (satisfying *τ*^*−1*^*·τ* *=* *l*). Let *π* = *τ*^*−1*^*·σ*, then the inversion distance from *τ* to *σ* is transformed into *d*_*(π,l)*_ of the inversion distance from *π* to *l*. So, next we will study the distance between any permutation *π* and the identity permutation *l*.

In order to deal with the data at both ends of permutation, we insert *π*_0_ = 0, *π*_n+1_ = *n* + 1 at both ends of permutation *π*, and call *π*=(0, *π*_1_, *π*_2_, *π*_3_,…, *π*_*n*,*n*+1_) extension permutations.

In the extension arrangement, if *π*_*i*_ and *π*_*i+1*_ are adjacent numbers (0 ≤ *i* ≤ *n*), then *π*_*i*_ and *π*_*i+1*_ are adjacency; otherwise, *π*_*i*_ and *π*_*i+1*_ are breakpoints. In this paper, the interval between two adjacent breakpoints in *π* is defined as a strip, that is, the largest fragment without a breakpoint. The further differentiation of strip can be divided into ascending strip and descending strip. The strip with only one element can be defined as either an ascending strip or descending strip, but it is conventionally defined as a descending strip (0 element and *n* + 1 element are always defined as ascending strip).

For example, in the extension arrangement *π = *(0, 2, 1, 3, 4, 5, 8, 7, 6, 9), there are 4 breakpoints in total, which are (0, 2), (1, 3), (5, 8), and (6, 9); there are 5 pairs of adjacent, respectively, (2, 1), (3, 4), (4, 5), (8, 7), and (7, 6); and there are 2 descending strips, respectively, (2, 1), (8, 7, 6), and 3 ascending strips, respectively 0, (3, 4, 5), 9.

The identity permutation does not contain any breakpoints, so in order to convert *π* into *l*, the breakpoints in *π* should be eliminated after the least number of reversals.

It has been proved that if the gene has direction, the reverse genome rearrangement problem is polynomial time solvable, and a very effective algorithm has been found. However, if the gene is unsigned, the reverse genome rearrangement problem is NP hard [5, 6]. In this paper, we mainly study the problem of unsigned reverse genome rearrangement. If there is no special explanation below, genome rearrangement will mean the unsigned reverse genome rearrangement. In 1995, David Sankoff and Kececioglu began to study the inversion distance problem and discussed the greedy approximation algorithm based on breakpoint elimination and an accurate algorithm of the branch and bound algorithm for the first time [7]. Then, Afna and Pevzner designed a 1.75-fold approximation algorithm for genome inversion sequencing without symbol, with a time complexity of O (n^2^). In 1998, Christie gave a polynomial approximation algorithm with an approximation degree of 1.5 and a time complexity of O (n^4^) [8]. Berman et al. designed a polynomial approximation algorithm with an approximation degree of 1.375 by using the signed reverse sorting algorithm and the cycle decomposition approximation algorithm [9]. In the twentieth century, Professor Mo Zhongxi's team of Wuhan University designed a greedy algorithm based on breakpoint graph, and Professor Zhu Daming of Shandong University designed a greedy algorithm based on the First Descending Strip Reversal (FDSR) [10]. Many researchers have developed various algorithms since then.

At present, the diversity and complexity of the reverse genome rearrangement algorithm make it impossible for many users to choose the algorithm suitable for different DNA sequence characteristics, which leads to unnecessary errors in the research process. On the other hand, it is difficult to understand the structure of the reverse genome rearrangement algorithm, which will affect the correct use of the algorithm in the actual situation. Because of the low abstraction of the reverse genome rearrangement algorithm, the reusability and reliability of the reverse genome rearrangement software are affected. Therefore, it is necessary to study the reverse genome algorithm at the domain level. The research on the algorithm family is helpful to extract the commonness and variability of the algorithm and provide support for the formal development of the reverse genome rearrangement algorithm.

### 2.2. Feature Modeling Technology

Domain modeling needs to determine key concepts and feature modeling of key concepts [11]. Feature engineering [12] holds that feature is a first-order entity that runs through the software life cycle, spans the problem space and solution space, and reduces the difference in demand awareness between users and software developers through features. In FODA [13], features are regarded as aspects, qualities, characteristics, and so forth that are visible, obvious, or characteristic to users in software systems. Features are domain knowledge accumulated by users' experts after long-term use or research in a domain.

Feature modeling is the activity of modeling the commonality and variability of features and the relationship between them. Literature [14] puts forward a feature-oriented domain modeling method (FODM), which considers the characteristics of service, function, and behavior of the domain and obtains the feature model through service analysis activities, function analysis activities, behavior analysis activities, domain terminology analysis activities, common variability analysis activities, interactive process analysis activities, and quality demand analysis activities.

### 2.3. Formal Method PAR

The Par [15–19] (partition and recur) method is a unified algorithm programming method based on partition and recur. It makes full use of mature programming technologies such as data abstraction, function abstraction, software reuse, and class genus, to realize the formal development of complex algorithm problems. That is, through a series of formal transformations to the problem specification, a fast and correct algorithm is obtained, and then an executable language program is obtained through a series of formal equivalent transformations or software conversion tools. It consists of the following elements: SNL (structured natural language), Radl (recurrence based algorithm design language), APLA (Abstract Programming Language), a set of model transformation rules, and a set of automatic conversion tools and executable programs among requirements model, algorithm model, and abstract program model. The APLA language fully embodies modern programming ideas such as function abstraction and data abstraction, which make it very suitable for describing abstract algorithm programs. In APLA, all the combined data types and their related operations adopt the generic mechanism. The generics are mainly divided into two categories: ① type parameterization, the introduction of the keyword sometype, which can be used to define type variables, and the basic type of the combined data type can be directly described in the form of parameters in the type declaration and ② subroutine parameterization: the func and proc keywords are provided in APLA to declare the process parameters and function parameters. When declaring these parameters, you only need to define the operation contains several variables and the type of each variable, and it can be instantiated by taking a subroutine implementation as argument. Apla is not only the target language of Radl-Apla program converter but also the source language of Apla to Ada, Java, *C*++, Python, and other executable language program converters, which is beneficial to the formal development of reusable components.

## 3. Domain Analysis and Abstraction of Genome Rearrangement Algorithm

### 3.1. Domain Analysis

Here, we deeply analyze the core ideas of three typical greedy algorithms.

#### 3.1.1. FDSR Algorithm

FDSR algorithm is a greedy algorithm developed by Zhu Daming, a teacher from Shandong University, with an approximate degree of 1.5 and a time complexity of O(n2). Its main process can be summarized as follows:

① Input a gene permutation *π* to judge the validity of gene arrangement. If it is not legal, the output is wrong. ② The extended *π* is an extension arrangement, *π*=(0, *π*_1_, *π*_2_, *π*_3_,…, *π*_*n*,*n*+1_), and the inversion distance *d* is set to 0. ③ Judge whether *π* is the identity permutation; if not, enter into ④. If it is, enter ⑨. ④ If the first strip other than strip 0 is ascending, it is reversed to a descending strip. ⑤ Find the position *i* of the smallest term (i.e., the last term) in the first descending strip and the position *j* of its inverse adjacent element. ⑥ If the inverse adjacent element is the first element of a descending strip, the strip where the inverse adjacent element is located is first flipped. ⑦ If the position of *j* is on the right side of *i*, the inversion interval is *ρ* = [*i* + 1, j] and if the position of *j* is on the left side of *i*, the inversion interval is *ρ* = [i, *j* + 1]. ⑧ Let *π* = *πρ*, increase the inversion distance *d* by 1 and return to ③. ⑨ Output reverse distance *d*.

#### 3.1.2. Algorithm Based on Breakpoint Graph

The algorithm based on breakpoint graph is a greedy algorithm with time complexity O (max{b3 (*π*), nb (*π*)}) and space complexity O (*n*), which is developed by Mo Zhongxi's team of Wuhan University. Its main process is as follows:

① Input the extension permutation *π* and judge whether *π* is legal; if not, end. Then, judge whether it is the identity permutation. If it is, end, otherwise, determine the inverse permutation *π*^*−1*^ of *π* and the breakpoint set *B*_*π*_ of *π*, *π*′s breakpoint location table T. Let *i* = 1.

② Based on the breakpoint location table, find out all the reverse intervals in *π* that can eliminate two breakpoints and one breakpoint, and store them in S2 and S1, respectively.

③ If *S*_*2*_ is empty, enter ④. Otherwise, find a reverse interval *ρ* from *S*_*2*_, so that *πρ* contains the largest number of descending strips. Let *ρ*_*i*_ *=* *ρ*, *b* (*π*) *=* *b* (*π*)*−*2; enter into ⑥. ④ If S1 is empty, enter into ⑤. Otherwise, select a reverse interval *ρ* from S1, so that *πρ* contains the largest number of descending strips; let *ρ*i = *ρ*, b (*π*) = *b* (*π*)−1, enter into ⑥. ⑤ Any reverse interval *ρ*i = [*m*, *n*] (*m* + 1 <*n*, *m* is the right end position of a breakpoint, and *n* is the left end position of a breakpoint). ⑥ Do reverse operation: let *π* = *πρ*, and correct *π*-1 accordingly. ⑦ If *π* = *πρ* is the identity permutation, enter into ⑧. Otherwise, modify the breakpoint set location table; let *i* = *i* + 1, and enter ②. ⑧ Output *i*, *ρ*1, *ρ*2, *ρ*3,…, *ρn*.

#### 3.1.3. Algorithm Based on Eliminating Breakpoints

The algorithm based on eliminating breakpoints is a greedy algorithm with an approximate degree of 2 designed by David Sankoff and Kececioglu. The main process can be summarized as follows:

① Input the extension permutation *π*, judge the correctness of permutation, and calculate *π*-1, array down, and array up (array down and up can judge whether there are ascending and descending strip in a certain interval within O(1)). ② Find an inversion interval that can eliminate two breakpoints. ③ If there is no reverse interval *ρ* that can eliminate two breakpoints, find a reverse interval *ρ* that can eliminate one breakpoint and make the new arrangement after *πρ* have a descending strip. ④ If the above does not exist, then find an inversion interval that can eliminate a breakpoint. ⑤ If the above does not exist, find the inversion interval [*i*, *πi*−1], if *π*i≠i (*i* is the minimum position of subscript of element *π*i≠i).

The above five steps until *π* are the identity permutation.

According to the above analysis, we can use a unified flow chart to express the idea of each algorithm, as shown in Figure 1.

### 3.2. Domain Modeling

In the following, we will use the feature modeling method proposed by academician Mei Hong's team to conduct feature modeling on the URGRA domain and construct the feature model based on the characteristics of service, function, and behavior in the URGRA domain. The reverse manipulation service (reverse_mani) is the core service in this domain, and sequence validity check (seq_check), gene permutation storage table manipulation (perm_store_mani), greedy algorithm mode option (greedy_op), auxiliary permutation storage table manipulation (auxiliary_permu_mani), judging whether it is identity arrangement (is_sorted), and output are the main functions in this field. Where seq_check, perm_store_mani, greedy_op, output are required functions, auxiliary_permu_mani, is_sorted are optional functions, for greedy_op, Breakpoint_diagram_op, FDSR_op, and breakpoint_op are its behavior characteristics. For output, output_mode is its significant behavior characteristic, and there are three main behavior characteristics: inversion process output (procedure_op), inversion distance output (distance_op), and inversion interval output (interval_op). For auxiliary_permu_mani, break_store, *π*^*−1*^ and break_pos_store, and array of *π*^*−1*^, up and down, are behavior characteristics. Based on the above analysis, a feature model for this domain is constructed, as shown in Figure 2.

Different features in that feature model realize a complete domain feature model through interaction, and the interaction between the features in the feature model needs to be reflected by the constraints and dependency between the included features.

Therefore, aiming at the feature model established above, we design the feature interaction model in the URGRA domain.

Through the establishment of the URGRA feature model, it is analyzed that the algorithm mainly includes three characteristics of the change process: permutation_mani, greedy_op, and output. In addition, the input of the algorithm in this field is gene sequence, and the legitimacy of sequence information needs to be checked before algorithm execution. So, the major artifacts in this domain are the seq_check artifact, the perm_store_mani artifact, the greedy_op artifact, and the output artifact. Other features in the feature model are used as auxiliary components, and the interaction model of components is established according to the dependency between components, as shown in Figure 3.

Wherein, the nodes connected by solid lines represent the basic features that must be included in the URGRA domain, and the direction represented by the arrow represents the execution priority of the four features from high to low. The dotted arrows represent the associated operations required during algorithm assembly, such as the use of auxiliary storage table operations for greedy mode selection. The dotted line indicates the interaction between two features during the execution of the algorithm; for example, when using the inversion output feature, when selecting the permutation process, the distance, or the inversion interval output, the gene permutation storage table operation is required.

### 3.3. Type and Algorithm Component Design

Here, we further analyze the abovementioned interaction design model of the URGRA domain feature model and algorithm component and encapsulate them into two abstract data type (ADT) components and a reverse rearrangement algorithm component. By virtue of the high abstraction of the Apla program, good support for ADT, and easy formal derivation and correctness verification, we carry out the formal design and implementation of the URGRA model based on Apla code.

#### 3.3.1. Gene Permutation Storage Table Type Component

  define ADT perm_store(sometype elem);
   type perm_store = private;
   var
   distance: integer;
   permutation:array [0...n,elem];
   aux:auxiliary_permu;
  procedure init (var p: perm_store; permutation:array[0...n,elem]);
   function check (p:perm_store; permutation:array [0...n,elem]):Boolean;
   function isSorted (p:perm_store; permutation:array[0...n,elem]):Boolean;
   procedure setValue(p:perm_store; i:integer; permutation:array[0...n,elem]);
   function getValue (p:perm_store; permutation:array[0...n,elem]; i:integer): elem;
   procedure reversal(p:perm_store; permutation:array[0...n,elem]; *i*:integer; j:integer; aux:auxiliary_permu);
   procedure distance_mani(p:perm_store; distance: integer);
   procedure output (p:perm_store; permutation:array[0...n,elem] = NULL; distance:integer);
  enddef;

This generic ADT name is perm_store, which contains a type parameter elem, which can accept either integer or character types. type perm_store = private is the storage space specification, which specifies that the storage space used by this self-defined ADT is private. init(var p: perm_store; permutation: array[0 ... n, elem]) is used to dynamically allocate storage space and initialize it. check (p: perm_store; permutation: array[0...n, elem]) is to verify whether the gene sequence is correct. isSorted(p:perm_store; permutation:array[0...n,elem]) is to determine whether the permutation is the identity arrangement. setValue(p:perm_store; i:integer; permutation:array[0...n,elem]) and getValue(p:perm_store; permutation:array[0...n,elem]; i:integer) function is to set the element value and get the element value. output(p:perm_store; permutation:array[0...n,elem] = NULL; distance:integer) indicates the inversion distance, inversion process, and inversion interval of the output permutation, and only the inversion distance is output by default. reversal(p:perm_store; permutation:array[0...n,elem]; i:integer; j:integer; aux:auxiliary_permu) indicates the inversion of the permutation. distance_mani(p:perm_store; distance: integer) indicates the operation to reverse the distance. The operation of this self-defined ADT type specified in Apla should pass this self-defined ADT type as an argument to a function or procedure as an operation object, so the above operations have a variable *p* of type perm_store.

#### 3.3.2. Auxiliary Permutation Storage Table Type Component

  define ADT auxiliary_permu(someproc initialization_auxiliary (sometype:elem); n:integer)
   type permutation = private;
   procedure set_value(a:auxiliary_permu; i:integer);
   function get_value(a:auxiliary_permu; i:integer):elem;
  enddef

The ADT contains a procedure generic parameter someproc initialization_ auxiliary(sometype:elem) and an integer parameter *n*, so that the generic program can support instantiating different greedy algorithm modes. type permission_mani = private is a storage space description, which is used to describe that the storage space used by the self-defined ADT is private. procedure set_value(a:auxiliary_permu; i:integer) and function get_value(a:auxiliary_permu; i:integer) are to set and obtain element values.

#### 3.3.3. Reverse Rearrangement Algorithm Component

  procedure greedy_reverse(p:FDSR_permutation_mani; a: FDSR_auxiliary);
  begin
   if(p.check(p,permutation))⟶
   do (┐p.is_sorted(p,permutation))
   ⟶p.reversal(p,permutation,i,j,a);
   p.reverse_mani(p,diatance);
   od;
   fi;
   a.output(p,diatance);
  end

## 4. Development of FDSR Rearrangement Algorithm Based on ADT

### 4.1. Inverse Rearrangement Algorithm Based on FDSR

  program FDSR;
  procedure FDSR_auxiliary_initialization(integer);
  var
   i:integer;
   length:integer;
   symbol:char;
  begin
   open(D:\FDSR\sourcedata.txt)
   for each(*i* = 0; *i* ≤ 2^*∗*^length + 3; *i*++)
   ……//program code segment, omitted
  end;
  ADT FDSR_auxiliary:new auxiliary_permu(FDSR_auxiliary_initialization,1);
  ADT FDSR_permutation_mani:new permutation_mani(integer);
  FDSR_reverse():new Procedure greedy_reverse(FDSR_permutation_mani, FDSR_auxiliary);
  Var:
   p:FDSR_permutation_mani
   a:FDSR_auxiliary
  begin//main program code
   open(D:\FDSR\sourcedata.txt)
   foreach(*i* = 0; *i* ≤ 2^∗^length+3; *i*++)
   ……//program code segment, omitted
   FDSR_reverse(p,a);
  end;

### 4.2. The Apla Program Is Converted to C++

After assembling components based on the Apla language into the FDSR algorithm, because the Apla program cannot run directly, we use Apla-C++ conversion tool in the PAR platform to convert the Apla program into *C*++ code. Selected if......fi statement in Apla is converted into if......else statement in *C*++, and circular do......od statement corresponds to do......while statement in *C*++; ADTs with member variables and member functions are converted into classes in *C*++, such as ADT permutation_mani and ADT auxiliary_permu.

## 5. Results and Discussion

The computer is configured with AMD A10-7300 Radeon R6,10 Compute Cores 4C+6 G 1.90 GHz, 12 GB memory, and Window 7 operating system.

We used real data to carry out the inversion test. Both human and mouse chromosomes have the same gene fragments, totaling 193 genes. These genes are described as follows [20]:

### 5.1. Mouse Gene Arrangement

61 25 26 27 28 22 15 14 13 12 16 86 87 89 85 88 84 83 82 24 23 40 104 103 102 21 159 160 162 161 125 38 37 10 9 7 6 5 8 11 4 62 63 79 80 81 2 78 3 1 66 149 39 41 124 68 69 70 71 20 34 90 112 111 109 110 113 114 115 116 157 158 156 101 100 106 99 96 97 98 75 44 72 73 43 155 42 136 17 76 132 108 107 131 130 36 35 32 30 31 64 92 165 164 153 123 122 121 67 19 51 49 50 138 139 137 144 143 141 140 145 146 142 147 148 18 129 54 53 52 47 29 93 91 126 128 74 127 45 46 77 167 168 117 118 120 119 135 134 166 33 163 65 133 59 58 57 60 56 55 154 150 151 152 48 105 95 94 174 173 175 176 177 184 185 187 186 172 171 179 180 181 182 183 178 170 169 188 189 190 191 192 193.

### 5.2. Human Gene Arrangement

1 2 3 4 5 6 7 8 9 10 11 12 13 14 15 16 17 18 19 20 21 22 23 24 25 26 27 28 29 30 31 32 33 34 35 36 37 38 39 40 41 42 43 44 45 46 47 48 49 50 51 52 53 54 55 56 57 58 59 60 61 62 63 64 65 66 67 68 69 70 71 72 73 74 75 76 77 78 79 80 81 82 83 84 85 86 87 88 89 90 91 92 93 94 95 96 97 98 99 100 101 102 103 104 105 106 107 108 109 110 111 112 113 114 115 116 117 118 119 120 121 122 123 124 125 126 127 128 129 130 131 132 133 134 135 136 137 138 139 140 141 142 143 144 145 146 147 148 149 150 151 152 153 154 155 156 157 158 159 160 161 162 163 164 165 166 167 168 169 170 171 172 173 174 175 176 177 178 179 180 181 182 183 184 185 186 187 188 189 190 191 192 193.

Read the mouse gene arrangement from sourcedata.txt, then output the inversion result to targedata.txt, as shown in Figure 4.

The running time is shown in Figure 5.

The FDSR algorithm developed by the formal PAR method runs for 3 ms.

With the formal method PAR, we first accurately describe the functional specification of reverse genome rearrangement in Radl language and then develop loop invariants based on the new strategy of developing loop invariants. Then, we develop an Apla algorithm program based on the obtained algorithm specification and loop invariants, thus formally implementing perm_store, auxiliary_permu type components, and reverse rearrangement algorithm component. Finally, we use these three components and assemble the FDSR algorithm with the support of the PAR platform. Compared with some existing algorithms, our formal developed algorithm ensures the reliability and robustness of the algorithm program and improves the assembly flexibility of the assembly algorithm by means of component assembly, which is convenient for researchers to maintain and optimize.

## 6. Conclusions

Reverse genome rearrangement is a hot topic in bioinformatics research, and its implementation algorithm has been widely studied. Because of the flexibility of its algorithm design strategy, this kind of algorithm presents more diversity and complexity. In this paper, the generative programming technology is used to deeply analyze the field of reverse genome rearrangement algorithm based on greedy strategy, find out the common features and variable features, design highly abstract program components based on Apla language by using formal method PAR, and generate FDSR algorithm by automatically assembling components supported by PAR platform, thus improving the reliability and reusability of algorithm components and reducing the development cost. Our team has formally implemented the pairwise sequence alignment algorithm component library and the multiple sequence alignment algorithm component library [21, 22]. In the next step, the insertion, deletion, and replacement of single characters in sequence alignment will be taken into account, so as to develop corresponding components and expand the scope of assemblable algorithms, to better analyze biological similarity and homology.

## Figures and Tables

**Figure 1:** Flow chart of reverse genome rearrangement algorithm.

**Figure 2:** URGRA feature model.

**Figure 3:** Feature interaction model of the algorithm component.

**Figure 4:** Output results.

**Figure 5:** Formal development of the FDSR algorithm by the PAR method.

## Data Availability

The data used to support the findings of this study are available in [20].
